# Carvacrol and PPARγ agonist, pioglitazone, affects inhaled paraquat-induced lung injury in rats

This article has been retracted.

**DOI:** 10.1038/s41598-021-87546-8

**Published:** 2021-04-14

**Authors:** Fatemeh Amin, Arghavan Memarzia, Hamideh Kazemi Rad, Hamid Reza Kazerani, Mohammad Hossein Boskabady

**Affiliations:** 1 Research Institute of Basic Medical Sciences, Rafsanjan University of Medical Sciences, Rafsanjan, Iran; 2 Department of Physiology and Pharmacology, School of Medicine, Rafsanjan University of Medical Sciences, Rafsanjan, Iran; 3 Applied Biomedical Research Center, Mashhad University of Medical Sciences, Mashhad, Iran; 4 Department of Physiology, Faculty of Medicine, Mashhad University of Medical Sciences, Mashhad, Iran; 5 Department of Physiology, Faculty of Veterinary Medicine, Ferdowsi University of Mashhad, Mashhad, Iran

**Keywords:** Physiology, Risk factors

## Abstract

Exposed rats to normal saline and paraquat (PQ) aerosol as control and PQ group, rats exposed to PQ and treated with 20 and 80 mg/kg/day carvacrol, 5 and 10 mg/kg/day pioglitazone, low dose of pioglitazone + carvacrol and 0.03 mg/kg/day dexamethasone (Dexa) for 16 days after the end of PQ exposure were studied (n = 6 in each group). Lung pathological changes, tracheal responsiveness to methacholine and ovalbumin (OVA) as well as transforming growth factor beta (TGF-β) and interleukin (IL)-6 level in the lung tissue homogenize as well as TGF-β, IL-6, oxidant and antioxidant levels oxidant and antioxidants were increased in PQ group (*p* < 0.01 to *p* < 0.001). Lung pathological changes, tracheal responsiveness to methacholine and OVA as well as TGF-β, IL-6 oxidant and antioxidant levels were improved in all treated groups except lung pathological changes in treated group with low dose of pioglitazone (*p* < 0.05 to *p* < 0.001). The effects of low dose of pioglitazone and carvacrol alone were significantly lower than in the combination group of low dose of pioglitazone + carvacrol (*p* < 0.05 to *p* < 0.001). Carvacrol treatment improved inhaled PQ-induced lug injury similar to the effects of dexamethasone. The synergic effect of carvacrol and pioglitazone suggests PPAR-γ receptor mediated effects of carvacrol on inhaled PQ-induced lung injury.

## Introduction

Paraquat (PQ, -1, 1´-dimethyl-4, 4´-bipyridinium dichloride) is an herbicide^1^ for controlling various crops^2^, and causes high toxicity^3–5^ as well as lethal effects (30 mg/kg) in humans^6^. Inflammation and oxidative stress, generation of intracellular reactive oxygen species, lipid peroxidation, and redox reactions of cellular membranes^7^ as well as increased interleukins and tumor necrosis factor alpha (TNF-α) in the lungs have been shown for PQ poisoning^8^. In farmers, PQ is usually absorbed in the lung tissue and causes leukocytosis, pulmonary inflammation, pneumonia, lung fibrosis, pulmonary hypertension, heart enlargement, acute renal damage, edema, increased serum levels of amylase, glucose, and creatinine^8^. Chronic exposure to PQ also induces alveolitis, inflammatory cell infiltration, and collagen deposition in the lung^9^. Poisoning with PQ is treated by activated charcoal, anti-inflammatory, immunosuppressive, and antioxidants agents such as acetylcysteine and salicylate^7^ though they are not able to cure PQ poising fully, and as such new drugs are needed to prevent PQ-induced lung injury^2,10^.

Carvacrol, is the active component of various medicinal plants^11^, with anti-inflammatory^12–17^, anti-oxidant, and immunomodulatory properties^18^. In addition, studies have also reported improvement of tracheal responsiveness, inflammatory mediators, and total plus differential WBC^12^, serum cytokines and endothelin levels^13^, and lung pathological changes, immunoglobulin E (IgE) and eosinophil peroxidase levels in the BALF^14^, serum levels of total protein, in guinea pigs model of asthma as well as various cytokine gene expressions^15^ and T helper cells subtypes along with their cytokine gene expression^16^ in the splenocytes of asthmatic mice with carvacrol treatment.

Anti-inflammatory and anti-cancer effects on lung diseases, pain, and obesity have been shown for peroxisome proliferator-activated receptors (PPARs)^19,20^ The regulations of cellular metabolism, cell differentiation, apoptosis, and inflammation^21–23^ have also reported by PPARγ ligands such as prostaglandins, leukotrienes, rosiglitazone, and pioglitazone^24^.

The aims of the present study are exploring the potential effects of carvacrol and PPARγ agonist (pioglitazone) on the lung injury induced by inhaled PQ and their possible synergic effects in male Wistar rats.

## Results

### Lung weight changes due to inhaled PQ and the effects of treatments

The lung’s wet and dry weights significantly increased in the animals exposed to inhaled PQ compared to the control group (*p* < 0.01 for wet and *p* < 0.05 for dry weight), (Fig. 1A, B). The lung’s wet weight significantly decreased in all treated groups and lung dry weight only in groups treated with a combination of Pio-5 + C-20 and dexamethasone compared to the PQ group (*p* < 0.05 to *p* < 0.01), (Fig. 1A, B). The improvement in the lung’s wet weight in the group treated with a combination of Pio-5 + C-20 was significantly higher than in pio-5 group (*p* < 0.05), (Fig. 1A). However, the W/D ratio was not significantly different among the studied groups (Fig. 1C).

**Figure 1:** Comparisons of lung wet (**A**) and dry (**B**) weight and wet/dry weight ratio (W/D) of the lung (**C**) between control group (Ctrl), group exposed to paraquat aerosol at doses of 54 mg/m^3^ (PQ-54 mg/m^3^), groups exposed to PQ-54 mg/m^3^ and treated with 5 and 10 mg/kg/day pioglitazone (Pio-5 mg/kg/day and Pio-10 mg/kg/day), 20 and 80 mg/kg/day carvacrol (C-20 mg/kg/day and C-80 mg/kg/day), 0.03 mg/kg/day dexamethasone (Dexa-0.03 mg/kg/day) and 5 mg/kg/day pioglitazone + 20 mg/kg/day carvacrol (Pio-5 mg/kg + C-20 mg/kg). +*p* < 0.05 compared to the PQ-54 mg/m^3^, #*p* < 0.05 compared to dexamethasone, £*p* < 0.0 comparisons between Pio-5 with Pio-5 mg/kg/day + C-20 mg/kg/day group. Data are presented as mean ± SEM (n = 6 in each group). Comparisons between different groups were made using one-way ANOVA followed by Tukey’s multiple comparison test.

### Lung pathological changes due to inhaled PQ and the effects of treatments

The lung’s pathological changes including interstitial inflammation, edema, interstitial fibrosis, and emphysema significantly increased in the group exposed to inhaled PQ (*p* < 0.001 for all cases, Fig. 2). In all treated groups, all lung pathological variables significantly improved compared to the PQ group except Pio-5 for all variables and C-20 for lung edema and interstitial fibrosis (*p* < 0.05 to *p* < 0.001, Fig. 2). The improvements in lung edema in C-20 and Pio-5 groups and that of interstitial fibrosis in C-20, Pio-5, and Pio-10 groups were significantly lower than in Dexa-0.03 group (*p* < 0.001 for interstitial fibrosis and *p* < 0.05 for other cases, Fig. 2). The improvement in all pathological changes in C-20 and Pio-5 groups were significantly lower than the combination therapy of Pio-5 + C-20 groups (*p* < 0.05 to *p* < 0.001, Fig. 2). A photograph specimen of the lung in each studied group is shown in Fig. 3.

**Figure 2:** Comparisons of emphysema (**A**), interstitial inflammation (**B**), edema (**C**) and interstitial fibrosis (**D**) between control group (Ctrl), group exposed to paraquat aerosol at doses of 54 mg/m^3^ (PQ-54 mg/m^3^), groups exposed to PQ-54 mg/m^3^ and treated with 5 and 10 mg/kg/day pioglitazone (Pio-5 mg/kg/day and Pio-10 mg/kg/day), 20 and 80 mg/kg/day carvacrol (C-20 mg/kg/day and C-80 mg/kg/day), 0.03 mg/kg/day dexamethasone (Dexa-0.03 mg/kg/day) and 5 mg/kg/day pioglitazone + 20 mg/kg/day carvacrol (Pio-5 mg/kg + C-20 mg/kg). ***p < 0.001 compared to the control group. +*p* < 0.05, ++*p* < 0.01, and +++*p* < 0.001 compared to PQ-54 mg/m^3^, #*p* < 0.05 and ###*p* < 0.001 compared to dexamethasone, $*p* < 0.05 compared to Pio-5 mg/kg/day, £*p* < 0.05, ££*p* < 0.01and £££*p* < 0.001 comparison between C-20 and Pio-5 with Pio-5 mg/kg/day + C-20 mg/kg/day group. Data are presented as mean ± SEM (n = 6 in each group). Comparisons between different groups were made using one-way ANOVA followed by Tukey’s multiple comparison test.

**Figure 3:** Lung specimens photographs of the control group (Ctrl), group exposed to paraquat aerosol at doses of 54 mg/m^3^ (PQ-54 mg/m^3^), groups exposed to PQ-54 mg/m^3^ and treated with 5 and 10 mg/kg/day pioglitazone (Pio-5 mg/kg/day and Pio-10 mg/kg/day), 20 and 80 mg/kg/day carvacrol (C-20 mg/kg/day and C-80 mg/kg/day), 0.03 mg/kg/day dexamethasone (Dexa-0.03 mg/kg/day) and 5 mg/kg/day pioglitazone + 20 mg/kg/day carvacrol (Pio-5 mg/kg + C-20 mg/kg)., (Magnification: 10 × 20).

### Tracheal responsiveness changes due to inhaled PQ and the effects of treatments

Methacholine cumulative dose response curve in the group exposed to inhaled PQ was shifted to the right compared to the control group (Fig. 4A). The value of EC_50_ in the group exposed to inhaled PQ was significantly lower than in the control group (*p* < 0.001, Fig. 5A).

**Figure 4:** Cumulative concentration response curves to methacholine in the control group (Ctrl) and group exposed to paraquat aerosol at doses of 54 mg/m^3^ (PQ-54 mg/m^3^), (**A**) PQ-54 mg/m^3^, groups exposed to PQ-54 mg/m^3^ and treated with 10 mg/kg/day pioglitazone (Pio-10 mg/kg/day), 80 mg/kg/day carvacrol (C-80 mg/kg/day) and 0.03 mg/kg/day dexamethasone (Dexa-0.03 mg/kg/day), (**B**) and groups exposed to PQ-54 mg/m^3^ and treated with 5 mg/kg/day pioglitazone (Pio-5 mg/kg/day), 20 mg/kg/day carvacrol (C-20 mg/kg/day) and 5 mg/kg/day pioglitazone + 20 mg/kg/day carvacrol (Pio-5 mg/kg + C-20 mg/kg), (**C**).

**Figure 5:** Comparisons of concentration of methacholine causing 50% maximum contractile response of tracheal smooth muscle to methacholine (EC_50_) (**A**), and tracheal contractile response to ovalbumin (OVA), (**B**) between control group (Ctrl), group exposed to paraquat aerosol at doses of 54 mg/m^3^ (PQ-54 mg/m^3^), groups exposed to PQ-54 mg/m^3^ and treated with 5 and 10 mg/kg/day pioglitazone (Pio-5 mg/kg/day and Pio-10 mg/kg/day), 20 and 80 mg/kg/day carvacrol (C-20 mg/kg/day and C-80 mg/kg/day), 0.03 mg/kg/day dexamethasone (Dexa-0.03 mg/kg/day) and 5 mg/kg/day pioglitazone + 20 mg/kg/day carvacrol (Pio-5 mg/kg + C-20 mg/kg). ***p < 0.001 compared to the control group. ++*p* < 0.01, and +++*p* < 0.001 compared to PQ-54 mg/m^3^, #*p* < 0.05 compared to dexamethasone, $*p* < 0.05 compared to C-20 mg/kg/day, £*p* < 0.05 comparison between Pio-5 and C-20 with Pio-5 mg/kg/day + C- 20 mg/kg/day group. Data are presented as mean ± SEM (n = 6 in each group). Comparisons between different groups were made using one-way ANOVA followed by Tukey’s multiple comparison test.

On the other hand, methacholine cumulative dose response curves in all treated groups were shifted to the right compared to the PQ exposed group (Fig. 4B). The values of EC_50_ in all treated groups were significantly higher than in the PQ (*p* < 0.001 for all cases, Fig. 5A). In addition, methacholine cumulative dose response curves in Pio-5 and C-20 were shifted to the left compared to that of the Pio-5 + C-20 combination group (Fig. 4C). The value of EC_50_ in C-20 was also significantly lower than in the Pio-5 + C-20 combination group (*p* < 0.05, Fig. 5A).

Tracheal responsiveness to OVA was significantly increased in the group exposed to inhaled PQ as compared to the control group (*p* < 0.001, Fig. 5B).

In all treated groups, tracheal responsiveness to OVA was significantly improved compared to the PQ exposed group (*p* < 0.01 for C-20 and Pio-5 and *p* < 0.001 for other groups, Fig. 5B). Tracheal responsiveness to OVA was significantly lower in C-80 than its smaller dose (C-20) and Dex 0.05 (*p* < 0.01 for both cases Fig. 5B). Tracheal responsiveness to OVA was also higher in Pio-5 than in the Pio-5 + C-20 combination group (*p* < 0.05, Fig. 5A).

### Transforming growth factor beta and Interleukin 6 levels changes due to inhaled PQ and the effects of treatments

The levels of TGF-β and Interleukin (IL)-6 in the homogenized lung tissue were increased in the group exposed to inhaled PQ compared to the control group (*p* < 0.001 for both cases, Figs. 6 and 7).

**Figure 6:** Comparison of transforming growth factor beta (TGF-β) between control group (Ctrl), group exposed to paraquat aerosol at doses of 54 mg/m^3^ (PQ-54 mg/m^3^), groups exposed to PQ-54 mg/m^3^ and treated with 5 and 10 mg/kg/day pioglitazone (Pio-5 mg/kg/day and Pio-10 mg/kg/day), 20 and 80 mg/kg/day carvacrol (C-20 mg/kg/day and C-80 mg/kg/day), 0.03 mg/kg/day dexamethasone (Dexa-0.03 mg/kg/day) and 5 mg/kg/day pioglitazone + 20 mg/kg/day carvacrol (Pio-5 mg/kg + C-20 mg/kg). ***p < 0.001 compared to the control group. ++*p* < 0.01, and +++*p* < 0.001 compared to the PQ-54 mg/m^3^, #*p* < 0.05 and ##*p* < 0.01 compared to dexamethasone, $*p* < 0.05 compared to Pio-5 mg/kg/day, £££*p* < 0.001comparison between Pio-5 and C-20 with Pio-5 mg/kg/day + C-20 mg/kg/day group. Data are presented as mean ± SEM (n = 6 in each group). Comparisons between different groups were made using one-way ANOVA followed by Tukey’s multiple comparison test.

**Figure 7:** Comparison of IL-6 level between control group (Ctrl), group exposed to paraquat aerosol at doses of 54 mg/m^3^ (PQ-54 mg/m^3^), groups exposed to PQ-54 mg/m^3^ and treated with 5 and 10 mg/kg/day pioglitazone (Pio-5 mg/kg/day and Pio-10 mg/kg/day), 20 and 80 mg/kg/day carvacrol (C-20 mg/kg/day and C-80 mg/kg/day), 0.03 mg/kg/day dexamethasone (Dexa 0.03 mg/kg/day) and 5 mg/kg/day pioglitazone + 20 mg/kg/day carvacrol (Pio-5 mg/kg + C-20 mg/kg). ***p < 0.001 compared to the control group. +*p* < 0.05, ++ *p* < 0.01, and +++*p* < 0.001 compared to the PQ-54 mg/m^3^, £*p* < 0.05comparison between Pio-5 and C-20 with Pio-5 mg/kg/day + C-20 mg/kg/day group. Data are presented as mean ± SEM (n = 6 in each group). Comparisons between different groups were made using one-way ANOVA followed by Tukey’s multiple comparison test.

In all treated groups, TGF-β level was significantly reduced compared to the PQ exposed group (*p* < 0.01 for C-20 and Pio-5 and *p* < 0.001 for other groups, Fig. 6). The level of TGF-β in C-20, C-80, and Pio-5 was significantly higher than in the dexamethasone treated group (*p* < 0.05 to *p* < 0.01, Fig. 6). In the Pio-5 group, TGF-β level was significantly higher than in the Pio-10 group (*p* < 0.05, Fig. 6). The level of TGF-β in Pio-5 and C-20 groups was also higher than in the Pio-5 + C-20 combination group (*p* < 0.001 for both cases, Fig. 6).

In the groups treated with the high dose of carvacrol and pioglitazone as well as dexamethasone and the combination of low dose carvacrol and pioglitazone, IL-6 level was significantly reduced compared to the PQ exposed group (*p* < 0.05 to *p* < 0.001, Fig. 7). The level of IL-6 was significantly higher in the C-20 group than in the Pio-5 + C-20 combination group (*p* < 0.01, Fig. 7).

### Oxidative stress markers due to inhaled PQ and the effects of treatments

The levels of all oxidant and antioxidant biomarkers were significantly deteriorated in the bronchoalveolar lavage fluid (BALF) of inhaled PQ group compared to the control group (*p* < 0.01 for SOD and thiol and *p* < 0.001 for other cases, Figs. 8 and 9).

**Figure 8:** Comparison of MDA (**A**) and NO_2_ (**B**) levels between control group (Ctrl), group exposed to paraquat aerosol at doses of 54 mg/m^3^ (PQ-54 mg/m^3^), groups exposed to PQ-54 mg/m^3^ and treated with 5 and 10 mg/kg/day pioglitazone (Pio-5 mg/kg/day and Pio-10 mg/kg/day), 20 and 80 mg/kg/day carvacrol (C-20 mg/kg/day and C-80 mg/kg/day), 0.03 mg/kg/day dexamethasone (Dexa-0.03 mg/kg/day) and 5 mg/kg/day pioglitazone + 20 mg/kg/day carvacrol (Pio-5 mg/kg + C-20 mg/kg). ***p < 0.001 compared to the control group. +*p* < 0.05, ++*p* < 0.01, and +++*p* < 0.001 compared to the PQ-54 mg/m^3^, ##*p* < 0.01 compared to dexamethasone, $$*p* < 0.01 compared to Pio-5 mg/kg/day, £*p* < 0.05 and £££*p* < 0.001comparison between Pio-5 and C-20 with Pio-5 mg/kg/day + C-20 mg/kg/day group. Data are presented as mean ± SEM (n = 6 in each group). Comparisons between different groups were made using one-way ANOVA followed by Tukey’s multiple comparison test.

**Figure 9:** Comparison of SOD (**A**) CAT (**B**) activates and tiol (**C**) between control group (Ctrl), group exposed to paraquat aerosol at doses of 54 mg/m^3^ (PQ-54 mg/m^3^), groups exposed to PQ-54 mg/m^3^ and treated with 5 and 10 mg/kg/day pioglitazone (Pio-5 mg/kg/day and Pio-10 mg/kg/day), 20 and 80 mg/kg/day carvacrol (C-20 mg/kg/day and C-80 mg/kg/day), 0.03 mg/kg/day dexamethasone (Dexa-0.03 mg/kg/day) and 5 mg/kg/day pioglitazone + 20 mg/kg/day carvacrol (Pio-5 mg/kg + C-20 mg/kg). **p < 0.01 and ***p < 0.001 compared to the control group. +*p* < 0.05, ++*p* < 0.01, and +++*p* < 0.001 compared to the PQ-54 mg/m^3^, #*p* < 0.05, ##*p* < 0.01 and ###*p* < 0.001 compared to dexamethasone, $$*p* < 0.01 compared to Pio-5 mg/kg/day, £*p* < 0.05, ££*p* < 0.01 and £££*p* < 0.001comparison between Pio-5 and C-20 with Pio-5 mg/kg/day + C-20 mg/kg/day group. Data are presented as mean ± SEM (n = 6 in each group). Comparisons between different groups were made using one-way ANOVA followed by Tukey’s multiple comparison test.

The NO_2_ level was significantly decreased in all treated groups as well as MDA level in the groups treated with the high dose of carvacrol and pioglitazone as well as dexamethasone and combination of low dose carvacrol and pioglitazone, as compared to the PQ group (*p* < 0.05 to *p* < 0.001, Fig. 8). However, the levels of all anti-oxidant markers (CAT, SOD and thiol) were significantly increased in the BALF of the groups treated with the high dose of carvacrol and pioglitazone as well as dexamethasone and Pio-5 + C-20 combination (*p* < 0.05 to *p* < 0.001, Fig. 9). The effect of high dose pioglitazone on MDA, SOD, and CAT levels was significantly higher than its low concentration (*p* < 0.05 for SOD and *p* < 0.01 for other cases, Figs. 8 and 9).

The values of oxidant and antioxidant biomarkers in all treated groups were significantly improved compared to the PQ group (*p* < 0.05 to *p* < 0.001, Figs. 8 and 9). The effect of low dose carvacrol on NO_2_ level, the impact of low dose pioglitazone on MDA, SOD, and CAT levels, as well as the effects of both doses of carvacrol and pioglitazone were significantly lower than the dexamethasone treated group (*p* < 0.05 to *p* < 0.001, Figs. 8 and 9).

## Discussion

This study was designed to evaluate the effects of carvacrol, pioglitazone, and pioglitazone + carvacrol combination on lung injury induced by inhaled PQ along with the possible mechanisms of these effects. The lung’s wet and dry weight, lung histology, tracheal responsiveness to methacholine, and OVA as well as TGF-β, IL-6, oxidants, and antioxidants levels were deteriorated in the group exposed to PQ. These results indicate induction of lung injury by inhaled PQ through inflammatory and oxidative stress processes, lung pathological changes and increased tracheal responsiveness to methacholine and OVA.

The PQ dose used in the present study was chosen according the only study that had examined the effect of inhaled PQ at doses of 0.83–2.07 mg/m^3^^25^ so far. Nevertheless, the exposure time period in each session decreased while the duration of exposure and PQ dose increased. The duration of the study was also chosen based on several previous studies reporting increased tracheal responsiveness to methacholine, cell count, interleukin 17 (IL-17), TGF-β levels in the BALF, and collagen deposition in the lung 15 days following PQ administration in mice^26^, induced lung pathological changes 28 days after PQ administration in Wistar rats^27^, and increased W/D of lung weight ratio, lung fibrosis as well as diminished arterial oxygen partial pressure, 7, 14, 21, and 28 days following PQ administration^28^.

Several previous studies support the effects of PQ on the lung as observed in the current study. Increased total protein of the lung tissue and serious histopathological changes in the lung tissue were shown due to administration of 20 mg/kg, i.p PQ for 3 days^29^. Administration of PQ (15 mg/kg/mL, i.p.) increased lung fibrosis, transforming growth factor-1β (TGF-1β) and malondialdehyde (MDA) levels in the lung as well as neopterin and antioxidant levels in the serum^30^. Infiltration of inflammatory cells in the lung’s interstitial tissues^31^ and BALF, along with total and differential white blood cell (WBC)^32^ increased 48 h following a single dose (30 mg/kg) of PQ. Administration of PQ (10 mg/kg, i.p.) increased cellular recruitment, IL-17 and TGF-β levels in the BALF, collagen deposition in the lung and tracheal responsiveness to methacholine^26^. Lung pathological changes were also reported after administration of PQ for 2 weeks in rats^27^. Increased lymphocyte count, TNF-α, C-reactive protein (CRP), and retinol binding protein (RBP) levels were demonstrated in patients with acute PQ poisoning^33^. However, the effect of inhaled PQ on the lug was shown in this study which is the common way of exposing farmers to this toxin.

The main mechanisms of the effect of PQ on the lung have been suggested as the alveolar and Clara cell membrane expression of polyamine transport system expression as well as induction of lung inflammation and oxidative stress as reported previously^34^. Reduction of nicotinamide adenine dinucleotide phosphate (NADPH) levels, as membrane lipid peroxidation has also been reported to contribute to the PQ-induced lung injury^35^. Treatment with both doses of pioglitazone significantly decreased the lung’s wet weight, tracheal responsiveness to methacholine and OVA, as well as TGF-β and IL-6 levels, while the lung’s pathological changes were reduced only due to high doses of pioglitazone. The levels of oxidant biomarkers were reduced but those of antioxidants increased due to pioglitazone treatment. The effects of high dose pioglitazone on most variables were higher than the impacts of its low dose. The results of treatment of PQ exposed animals with pioglitazone, demonstrated reduction of lung pathological changes and tracheal responsiveness which could be due to the ameliorating effect of pioglitazone on inflammatory and oxidative stress processes.

Anti-inflammatory and antioxidant effects of pioglitazone and other PPAR-γ agonists are well documented which support the effects of pioglitazone on lung injury due to inhaled PQ in rats observed in the current study. Pioglitazone (1–30 mg/kg) inhibits increased myeloperoxidase activity as well as intestinal TNF-α protein and messenger RNA (mRNA) expression^36^. Pioglitazone could also improve the antioxidant capacity, and increase super oxide dismutase (SOD) and catalase (CAT) enzymes in a kidney ischemia–reperfusion model^37^. Increased interleukin 4 (IL-4), but decreased interferon gamma (IFN-γ), TNF-α, and interleukin 6 (IL-6) levels were reported via pioglitazone^38^. Treatment with the combination of pioglitazone (15 mg/kg/day) and metformin improved lung adenoma cancero^39^, reduced nitric oxide (NO), TNF-α, interleukin 1-beta (IL-1β), IL-6, and interleukin 8 (IL-8) but elevated IL-4 and interleukin10 (IL-10) levels in lipopolysaccharide stimulated astrocytes (LPS-stimulated astrocytes)^40^. Pioglitazone (10 μM, for 1 or 3 h) treatment also decreased degranulation and adhesion of neutrophils in LPS-induced lung injury^41^. Paraquat-induced pulmonary inflammation was also diminished by atorvastatin through PPARγ receptors^42^. In patients with metabolic syndrome^43^ and subjects with advanced diabetic nephropathy^44^, pioglitazone treatment reduced WBC counts indicating its anti-inflammatory effects.

Carvacrol treatment reduced the lung’s wet weight, pathological changes, tracheal responsiveness to methacholine and OVA as well as TGF-β and IL-6 levels compared to the PQ-exposed group. Carvacrol treatment also decreased oxidant biomarker levels, but increased those of antioxidants. All changes were more pronounced in the group treated with the higher dose of carvacrol than its low dose. Thus, treatment of animals exposed to inhaled PQ with carvacrol decreased lung pathological changes and tracheal responsiveness to methacholine and OVA. These findings indicated the effect of carvacrol on inflammatory and oxidative stress processes induced by inhaled PQ in rats.

Anti-inflammatory, antioxidant, and immunomodulatory effects of carvacrol on lung disorders have previously been shown, which support the findings of the present study. Treatment with carvacrol improved tracheal responsiveness, inflammatory mediators, total and differential WBC^12^, serum cytokine and endothelin levels^13^, and lung pathological changes, immunoglobulin E (IgE) and eosinophil peroxidase levels in the BALF^14^, serum levels of total protein, phospholipase A2 (Phospholipases A2) and histamine^45^ in a guinea pig model of asthma as well as genes expression of various cytokines^15^ and T helper cells subtypes along with their cytokine gene expression^16^ in and splenocytes of asthmatic mice. In a guinea pig model of chronic obstructive pulmonary disease (COPD), carvacrol improved tracheal responsiveness and lung pathological changes^17^, lung inflammation and oxidative stress^46^, as well as systemic inflammation^47^.

Carvacrol also improved wheezing, forced expiratory volume in 1 s (FEV1), and nitrite plasma levels^48^ as well as pulmonary function tests, respiratory symptoms, hematological indices, and high-sensitivity C-reactive protein^49^ in asthmatic patients. In patients with sulfur mustard-induced lung disorders, carvacrol treatment for 2 months improved hematological parameters, oxidant/antioxidant biomarkers, and pulmonary function tests^50^ as well as inflammatory mediators and respiratory symptoms^51^. The plant extract also decreased IL4 but increased IFN-γ level and elevated IFN-γ/IL4 ratio, indicating increased Th1/Th2 balance in in vitro and in vivo studies in animal models of asthma and pripheral blood mononuclear cells respectively^52^.

Treatment with low doses of pioglitazone (5 mg/kg/day) + carvacrol (20 mg/kg/day), which was the most interesting part of the results, significantly improved all measured variables compared to PQ exposed group. Indeed, low doses of pioglitazone and carvacrol showed the lowest and in some cases non-significant effects. In addition, the effect of the combination treatment group with Pio-5 + C-20 was higher in most measured variables than the effects of low doses of pioglitazone and carvacrol alone. This finding suggests a synergic effect between pioglitazone and carvacrol which may indicate PPAR-γ receptor-mediated effects of carvacrol on lung injury induced by inhaled PQ. This suggestion was supported by the results of a study reporting on the activation of PPAR receptors and inhibition of cyclooxygenase-2 (COX-2) pathway through treatment with carvacrol^53^. However, further studies examining the effect of carvacrol in the presence of PPAR-γ receptors’ antagonist are required to confirm this suggestion.

Dexamethasone, a known anti-inflammatory drug used as a positive control treatment, also improved all measured variables which were not significantly different effects of high doses of pioglitazone, carvacrol, and combination of low dose of pioglitazone + low dose of carvacrol. The results of dexamethasone treated group support the anti-inflammatory, antioxidant, and immunomodulatory mechanisms of the effect of carvacrol on lung injury induced by inhaled PQ in rats.

However, there were a number of limitations in the present study. To examine the effect of carvacrol on PPAR-γ receptor more precisely, its effect in the presence of a PPAR-γ receptor antagonist drug should be evaluated which should be done in further studies. In addition, the effect of carvacrol alone and in combination with pioglitazone should be examined on inflammatory and molecular parameters such as IL-1beta, TNF-alpha, Caspase-3, Bax, and p53.

Inhaled PQ-induced of lung injury through inflammatory and oxidative stress processes, lung pathological changes and increased tracheal responsivenes. However, carvacrol showed ameliorating effects on lug injury induced by inhaled PQ which was similar to the effects of PPAR-γ agonist, pioglitazone, and dexamethasone. In addition, carvacrol revealed a synergic effect with pioglitazone which suggests PPAR-γ receptor-mediated effects of this agent on lung changes induced by inhaled PQ. These results may suggest a therapeutic effect of carvacrol on lung injury induced by PQ in farmers.

## Methods

### Animals and experimental groups

Forty-eight male Wistar rats, weighing 200–250 g were purchased and maintained in the Animal House of Faculty of Medicine, Mashhad University of Medical Sciences (MUMS), Mashhad under standard conditions as outlined in the previous study^54^. The study was approved by the ethics committee of MUMS (code961202), and criteria outlined in the Guide for Care and Use of Laboratory Animals (NIH US publication 23–68 revised 1985; http://oacuod.nih.gov/regs/guide/guidex.htm) were followed. The study was also carried out in compliance with the ARRIVE guidelines. The rats were randomly divided into eight groups, as shown in Table 1.

**Table 1:** Different studied groups, their exposure to saline solution or paraquate aerosols as well as their treatments (n = 6 in each group).

Groups	Exposed agents	Dose	Treated agents	Dose
Ctrl	Saline	–	–	–
PQ	Paraquat	54 mg/m^3^	–	–
C-20	Paraquat	54 mg/m^3^	Carvacrol	20 mg/kg/day
C-80	Paraquat	54 mg/m^3^	Carvacrol	80 mg/kg/day
Pio-5	Paraquat	54 mg/m^3^	Pioglitazone	5 mg/kg/day
Pio-10	Paraquat	54 mg/m^3^	Pioglitazone	10 mg/kg/day
Pio-5 + C-20	Paraquat	54 mg/m^3^	Pioglitazone + Carvacrol	Pio-5 mg/kg/day + C- 20 mg/kg/day
Dexa-0.03	Paraquat	54 mg/m^3^	Dexamethasone	0.03 mg/kg/day

*PQ* paraquat, *C* carvacrol, *Pio* pioglitazone, *Ctrl* control.

### Exposure of animals to aerosols of paraquat or saline and treatment protocol

Animal were exposed to saline solution in the control group or PQ (Sigma Aldrich Co, China), 8 times (every other day), each time for 30 min (total exposure period was 16 days). In other groups, aerosols as described in previous study were applied using a nebulizer (Omron CX3, Japan, particle size 3–5 μm) with head exposed chamber dimensions 15 × 18 × 30 cm^34^.

Animals were treated with carvacrol (purity 90%, Ji’An HaiRui Natural Plant, China), (20 and 80 mg/kg BW/day)^13^, pioglitazones (Samisaz Pharmaceutical Company, Iran), (5 and 10 mg/kg BW/day)^42^, combinations of carvacrol (20 mg/kg BW/day) + Pio (5 mg/kg BW/day)^34^, and dexamethasone (Dexa) (Sigma, St. Louis, MO, Germany), (0.03 mg/kg KB/day)^34^, via gavage for 16 days after the end of PQ exposure period. The saline (5 ml) was gavaged to the control and PQ-exposed groups on days 16–32. Appropriate concentrations of carvacrol and pioglitazone were prepared through diluting them in saline using few drops of tween-80. At the end of the treatment period (day 32), the rats were anesthetized through intraperitoneal injection of ketamine (50 mg/kg) and xylazine (5 mg/kg)^55^ (Fig. 10).

**Figure 10:** Exposing animals to aerosols of inhaled PQ (54 mg/m^3^) 8 times (days 1, 3, 5, 7, 9, 11, 13, 15 and treatment of animals with the carvacrol, pioglitazone and dexamethasone for 16 days after the end of exposure period. Animal were sacrificed in day 32 and various variables were measured.

### Lung weight measurement

At the end of the treatment period (day 33), the lungs were removed and their wet weight were determined. The lungs were then dried at 60 °C for 48 h with their dry weighted measured. The wet-to-dry weight (W/D) ratio of the lungs was calculated^32^.

### Lung pathological evaluation

Pathological changes of the left lung (following animal scarification and removal of the lung) including interstitial inflammation, edema, interstitial fibrosis, and emphysema were examined and scored as previously described (no pathologic changes = 0, patchy changes = 1, local changes = 2, scattered changes = 3, and severe changes in most parts of the lung = 4)^56^.

### Measurement of tracheal responsiveness to methacholine and ovalbumin

The tracheal ring was prepared as described previously^57^. Tracheal responsiveness to methacholine hydrochloride (Sigma Chemical Ltd, UK) was evaluated using cumulative concentrations (log)-response curve to methacoline and measurement of its effective concentration causing 50% of maximum response (EC_50_) was calculated^58^. Tracheal responses to OVA was also measured according a previous study^58^.

### Cytokines measurement

Transforming growth factor beta (TGF-β) level in the lung tissue homogenize and IL-6 were measured by specific enzyme-linked immunosorbent assay (ELISA) kits (Hangzhou Eastbiopharm, Iran) according to the manufacturer’s technique^59^.

### Oxidants’ and antioxidants’ measurements

Bronchoalveolar lavage (BALF) was prepared by cannulating the trachea and through lavage of the right lung by injecting 1 ml phosphate-buffered saline (PBS) solution 5 times and aspiration after gentle lung lavage. Oxidative markers such as malondialdehyde (MDA) and nitrite (NO_2_) as well as antioxidant markers including superoxide dismutase (SOD) and catalase (CAT) activities plus thiol group (SH) levels were measured in BALF. For this purpose, 1.5 ml BALF was centrifuged at 2500 rmp for 10 min with the oxidant and anti-oxidants markers measured in the supernatant of BALF as previously describeed^30,33^.

### Data analysis

Data were analyzed by the one-way analysis of variance (ANOVA) followed by Tukey’s multiple comparison test and results were presented as mean ± SEM. Values of *p* < 0.05 were considered as statistically significance.

## Data Availability

The raw data are available by the corresponding author upon request.

## References

[1] Hu X, Liang Y, Zhao H, Zhao M (2019). Effects of AT-RvD1 on paraquat-induced acute renal injury in mice. Int. Immunopharmacol..

[2] Dinis-Oliveira R (2008). Paraquat poisonings: mechanisms of lung toxicity, clinical features, and treatment. Crit. Rev. Toxicol..

[3] Chen HW, Tseng TK, Ding LW (2009). Intravenous paraquat poisoning. Chin. Med. J..

[4] Dhananjayan V, Ravichandran B (2018). Occupational health risk of farmers exposed to pesticides in agricultural activities. Curr. Opin. Environ. Sci. Health..

[5] Kim SJ, Gil HW, Yang JO, Lee EY, Hong SY (2009). The clinical features of acute kidney injury in patients with acute paraquat intoxication. Nephrol. Dial. Transplant..

[6] Yoon SC (2009). Clinical outcome of paraquat poisoning. Korean. J. intern. med..

[7] Gawarammana IB, Buckley NA (2011). Medical management of paraquat ingestion. Br. J. Clin. Pharmacol..

[8] Zhao G (2016). The effect of resveratrol on paraquat-induced acute lung injury in mice and its mechanism. Zhonghua. Wei. Zhong. Bing. Ji. Jiu. Yi. Xue..

[9] Yan B, Chen F, Xu L, Xing J, Wang X (2017). HMGB1-TLR4-IL23-IL17A axis promotes paraquat-induced acute lung injury by mediating neutrophil infiltration in mice. Sci. Rep..

[10] Sun L, Yan PB, Zhang Y, Wei LQ, Li GQ (2018). Effect of activated charcoal hemoperfusion on renal function in patients with paraquat poisoning. Exp. Ther. Med..

[11] Sajed H, Sahebkar A, Iranshahi M (2013). Zataria multiflora Boiss. (Shirazi thyme)—an ancient condiment with modern pharmaceutical uses. J. Ethnopharmacol..

[12] Boskabady MH, Jalali S (2013). Effect of carvacrol on tracheal responsiveness, inflammatory mediators, total and differential WBC count in blood of sensitized guinea pigs. Exp. Biol. Med..

[13] Jalali S, Boskabady MH, Rohani AH, Eidi A (2013). The effect of carvacrol on serum cytokines and endothelin levels of ovalbumin sensitized guinea-pigs. Iran. J. Basic. Med. Sci..

[14] Boskabady MH, Tabatabaee A, Jalali S (2014). Potential effect of the extract of Zataria multiflora and its constituent, carvacrol, on lung pathology, total and differential WBC, IgE and eosinophil peroxidase levels in sensitized guinea pigs. J. Funct. Foods..

[15] Kianmehr M, Rezaei A, Boskabady MH (2016). Effect of carvacrol on various cytokines genes expression in splenocytes of asthmatic mice. Iran. J. Basic. Med. Sci..

[16] Kianmehr M, Rezaee A, Mahmoudi M, Ghorani V, Boskabady MH (2019). T helper cells subtypes and their cytokine gene expression affected by carvacrol in sensitized mice administered during sensitization period. J. Cell. Biochem..

[17] Gholami-Mahtaj L, Boskabady M, Mohamadian-Roshan N (2015). The effect of Zataria multiflora and its constituent, carvacrol, on tracheal responsiveness and lung pathology in guinea pig model of COPD. Phytother. Res..

[18] Khazdair MR, Ghorani V, Alavinezhad A, Boskabady MH (2018). Pharmacological effects of *Zataria multiflora* Boiss L. and its constituents focus on their anti-inflammatory, antioxidant, and immunomodulatory effects. Fundam. Clin. Pharmacol..

[19] Tyagi S, Gupta P, Saini AS, Kaushal C, Sharma S (2011). The peroxisome proliferator-activated receptor: a family of nuclear receptors role in various diseases. J. Adv. Pharm. Technol. Res..

[20] Youssef, J. & Badr, M. Z. PPARs: history and advances. Peroxisome Proliferator-Activated Receptors (PPARs). Springer. 1–6 (2013).10.1007/978-1-62703-155-4_123100221

[21] Ghaedi K (2000). PEX3 is the causal gene responsible for peroxisome membrane assembly–defective Zellweger syndrome of complementation group G. Am. J. Hum. Genet..

[22] Wang L (2014). Natural product agonists of peroxisome proliferator-activated receptor gamma (PPARγ): a review. Biochem. Pharmacol..

[23] Ohtera A (2015). Identification of a new type of covalent PPARγ agonist using a ligand-linking strategy. ACS. Chem. Biol..

[24] Fujiki Y, Okiumoto K, Kinoshita N, Ghaedi K (2016). Lessons from peroxisome-deficient chinese hamster ovary (cho) cell mutants. Biochim. Biophys. Acta..

[25] Burleigh-Flayer H, Alarie Y (1987). Concentration-dependent respiratory response of guinea pigs to paraquat aerosol. Arch. Toxicol..

[26] Da-silva M, R. (2018). Beneficial effects of ascorbic acid to treat lung fibrosis induced by paraquat. PLoS ONE.

[27] Lalruatfela P, Saminathan M, Ingole R, Dhama K, Joshi M (2014). Toxicopathology of paraquat herbicide in female wistar rats. Asian. J. Anim. Vet. Adv..

[28] Zhang X (2019). synthetic receptor as a specific antidote for paraquat poisoning. Theranostics..

[29] Rezayat M (1998). Attenuation of paraquat toxicity in mice. M. J. I. R. I.

[30] Toygar M (2015). The relation between oxidative stress, inflammation, and neopterin in the paraquat-induced lung toxicity. Hum. Exp. Toxicol..

[31] Harchegani AL, Hemmati AA, Nili-Ahmadabadi A, Darabi B, Shabib S (2017). Cromolyn sodium attenuates paraquat-induced lung injury by modulation of proinflammatory cytokines. Drug. Res..

[32] Liu MW (2014). Protective effect of Xuebijing injection on paraquat-induced pulmonary injury via down-regulating the expression of p38 MAPK in rats. BMC. Complement. Altern. Med..

[33] Meng Z (2019). The effects of ω-3 fish oil emulsion-based parenteral nutrition plus combination treatment for acute paraquat poisoning. Int. J. Med. Res..

[34] Heydari, M. *et al*. The effect of Zataria multiflora hydroalcoholic extract on memory and lung changes induced by rats that inhaled paraquat. *Nutr. Neurosci*. 1–14 (2019).10.1080/1028415X.2019.166817331583983

[35] Smith L (1987). Mechanism of paraquat toxicity in lung and its relevance to treatment. Hum. Toxicol..

[36] Naito Y, Takagi T, Matsuyama K, Yoshida N, Yoshikawa T (2001). Pioglitazone, a specific PPAR-γ ligand, inhibits aspirin-induced gastric mucosal injury in rats. Aliment. Pharmacol. Ther..

[37] Zou C (2013). Pioglitazone protects against renal ischemia-reperfusion injury by enhancing antioxidant capacity. J. Surg. Res..

[38] Shigenobu T, Ohtsuka T, Shimoda M (2019). The prevention of tracheal graft occlusion using pioglitazone: A mouse tracheal transplant model study. Transpl. Immunol..

[39] Seabloom DE (2017). Fixed-dose combinations of pioglitazone and metformin for lung cancer prevention. Cancer. Prev. Res..

[40] Qiu D, Li XN (2015). Pioglitazone inhibits the secretion of proinflammatory cytokines and chemokines in astrocytes stimulated with lipopolysaccharide. Int. J. Clin. Pharmacol. Ther..

[41] Grommes J, Mörgelin M, Soehnlein O (2012). Pioglitazone attenuates endotoxin-induced acute lung injury by reducing neutrophil recruitment. Eur. Respir. J..

[42] Malekinejad H, Khoramjouy M, Hobbenaghi R, Amniattalab A (2014). Atorvastatin attenuates the paraquat-induced pulmonary inflammation via PPARγ receptors: a new indication for atorvastatin. Pestic. Biochem. Phys..

[43] Szapary PO (2006). Effects of pioglitazone on lipoproteins, inflammatory markers, and adipokines in nondiabetic patients with metabolic syndrome. Arterioscler. Thromb. Vasc. Biol..

[44] Agarwal R (2006). Anti-inflammatory effects of short-term pioglitazone therapy in men with advanced diabetic nephropathy. Am. J. Physiol. Renal. Physiol..

[45] Boskabady MH, Jalali S, Yahyazadeh N, Boskabady M (2016). Carvacrol attenuates serum levels of total protein, phospholipase A2 and histamine in asthmatic guinea pig. Avicenna. J. Phytomed..

[46] Boskabady MH, Mahtaj LG (2015). Lung inflammation changes and oxidative stress induced by cigarette smoke exposure in guinea pigs affected by *Zataria multiflora* and its constituent, carvacrol. BMC. Complement. Altern. Med..

[47] Mahtaj LG, Feizpour A, Kianmehr M, Soukhtanloo M, Boskabady MH (2015). The effect of carvacrol on systemic inflammation in guinea pigs model of COPD induced by cigarette smoke exposure. Pharmacol. Rep..

[48] Alavinezhad A, Hedayati M, Boskabady MH (2017). The effect of Zataria multiflora and carvacrol on wheezing, FEV1 and plasma levels of nitrite in asthmatic patients. Avicenna. J. phytomed..

[49] Alavinezhad A, Khazdair MR, Boskabady MH (2018). Possible therapeutic effect of carvacrol on asthmatic patients: a randomized, double blind, placebo-controlled, Phase II clinical trial. Phytother. Res..

[50] Amin F, Memarzia A, Kazerani HR, Boskabady MH (2020). Carvacrol and Zataria multiflora influenced the PPARγ agonist effects on systemic inflammation and oxidative stress induced by inhaled paraquat in rat: a randomized double-blind clinical trial. IJBMS..

[51] Khazdair MR, Boskabady MH (2019). The effect of carvacrol on inflammatory mediators and respiratory symptoms in veterans exposed to sulfur mustard, a randomized, placebo-controlled trial. Respir. Med..

[52] Boskabady MH, Mehrjardi SS, Rezaee A, Rafatpanah H, Jalali S (2013). The impact of *Zataria multiflora* Boiss extract on in vitro and in vivo Th1/Th2 cytokine (IFN-γ/IL4) balance. J. Ethnopharmacol..

[53] Hotta M (2010). Carvacrol, a component of thyme oil, activates PPARα and γ and suppresses COX-2 expression. J Lipid Res..

[54] Amin F, Roohbakhsh A, Memarzia A, Kazerani H, Boskabady MH (2020). Paraquat-induced systemic inflammation and increased oxidative markers in rats improved by Zataria multiflora extract and carvacrol. Avicenna. J. Phytomed..

[55] Alemán-Laporte J (2020). Combination of ketamine and xylazine with opioids and acepromazine in rats: physiological changes and their analgesic effect analysed by ultrasonic vocalization. Lab. Anim..

[56] Saadat S (2019). Aminoguanidine affects systemic and lung inflammation induced by lipopolysaccharide in rats. Respir. Res..

[57] Memarzia A (2019). The contribution of beta-2 adrenergic, muscarinic and histamine (H1) receptors, calcium and potassium channels and cyclooxygenase pathway in the relaxant effect of Allium cepa L. on the tracheal smooth muscle. J. Ethnopharmacol..

[58] Ghorani V (2018). The effects of allium cepa extract on tracheal responsiveness, lung inflammatory cells and phospholipase A2 level in asthmatic rats. Iran. J. Allergy. Asthma. Immunol..

[59] Shakeri F, Boskabady MH (2017). Anti-inflammatory, antioxidant, and immunomodulatory effects of curcumin in ovalbumin-sensitized rat. BioFactors.

